# Assessment of current practices and perceived effectiveness of injectable polynucleotide for enlarged facial pores among cosmetic physicians: A survey‐based evaluation

**DOI:** 10.1111/srt.13738

**Published:** 2024-09-04

**Authors:** Dagyeong Lee, Hosung Choi, Kyounghun Yoo, Young Jin Park, Hyun Jun Park, Seung Min Oh, Gun Hyon Ji, Gong Chan Rah, Dong Wook Shin

**Affiliations:** ^1^ Department of Family Medicine Hallym University Dongtan Sacred Heart Hospital Hwaseong Republic of Korea; ^2^ Piena Aesthetic Clinic Seoul Republic of Korea; ^3^ Lumi Clinic Seoul Republic of Korea; ^4^ Obliv Clinic Incheon Republic of Korea; ^5^ Maylin Clinic Seoul Republic of Korea; ^6^ Gangnam ON Clinic Seoul Republic of Korea; ^7^ Yonseidongan Clinic Seoul Republic of Korea; ^8^ Robbin Clinic Seoul Republic of Korea; ^9^ Department of Family Medicine/Supportive Care Center Samsung Medical Center Sungkyunkwan University School of Medicine Seoul Republic of Korea; ^10^ Department of Clinical Research Design & Evaluation Samsung Advanced Institute for Health Science & Technology (SAIHST) Sungkyunkwan University Seoul Republic of Korea

**Keywords:** effectiveness, enlarged facial pores, polynucleotides, practice

## Abstract

**Background:**

Polynucleotides stimulate collagen formation and are used clinically to enhance elasticity. In this study, we investigated current practices and perceived effectiveness of polynucleotide injection treatment for enlarged facial pores among cosmetic physicians.

**Materials and Methods:**

A survey was developed to investigate clinicians’ use and effectiveness of polynucleotides in the treatment of enlarged facial pores. This survey was distributed to clinicians at the Korean Aesthetic Surgery & Laser Society Autumn Symposium.

**Results:**

A total of 407 physicians who used polynucleotides for enlarged facial pores were enrolled in the survey. Polynucleotides were used by 75.7%, 87.7%, and 72.2% of physicians for enlarged facial pores caused by excessive sebum production, reduced elasticity, and acne, respectively. Among those users, 81.4%, 83.8%, and 76.8% in those same categories, respectively, responded that polynucleotides were “very effective” or “effective.” Furthermore, most clinicians combined polynucleotides with microneedle radiofrequency as energy‐based devices and with botulinum toxin as injection therapy.

**Conclusion:**

This study highlights the widespread use and perceived efficacy of polynucleotide injection among cosmetic physicians in the Republic of Korea for enlarged facial pores due to excessive sebum production, reduced elasticity, and acne. Positive feedback from practitioners supports the benefits of using polynucleotides in enlarged facial pore treatment.

**Abbreviations**
BoNT: botulinum toxin
PDRN: polydeoxynucleotide
PN: polynucleotides
RF: radiofrequency

## 1 INTRODUCTION

“Facial pore” typically refers to a facial surface feature corresponding to enlarged pilosebaceous follicle openings.^1^ Although enlargement of facial pores has not been defined clinically yet, a previous study reported three morphological subtypes of facial pores as follows: visible pores ranging from 0.1 to 0.6 mm^2^, enlarged pores measuring 0.3 to 0.6 mm^2^, and embedded blackhead pores.^2^ The various causes of enlarged facial pores include excessive sebum production, reduced skin laxity around the pores, and acne.^3^ The enlargement of facial pores can be a major cosmetic concern. Therefore, reducing the size of facial pores is of interest in the cosmetic field. Treatment options include reducing sebum production, improving skin elasticity, and treating acne with oral/topical agents, light/laser therapy, or botulinum toxin injection.^3^

Polydeoxynucleotide (PDRN) is derived from the germ cells of rainbow trout (*Oncorhynchus mykiss*) or chum salmon (*Oncorhynchus keta*), and is a mixture of deoxyribonucleotides.^4^ PDRN has anti‐inflammatory properties, as it can bind to the adenosine A2A receptor at the molecular level.^5^ A previous preclinical study has shown that PDRN stimulates new collagen formation and extracellular matrix protein synthesis.^6^ High‐molecular‐weight chained PDRNs are thought to primarily increase in the metabolic activity of fibroblasts,^7^ which are the main cells controlling renewal of various dermal components.

Polynucleotides (PN) is a bi‐polymer composed of 13 or more nucleotide monomers covalently bonded in a chain.^8^ PN is formed through controlled depolymerization, resulting in high molecular weight and a viscoelastic texture.^9^ Although its precise mechanism of action remains incompletely understood, the structural similarities between PN and PDRN are interesting. Consequently, the results of preclinical and clinical studies on PDRN may also be applicable to PN.

Many prior clinical studies have shown PN to be safe and effective for skin regeneration.^8^, ^10^, ^11^, ^12^ The use of PN in skin rejuvenation is mainly based on wound healing and regeneration, protection of the skin barrier, hydration, vascular stabilization, and anti‐inflammation.^13^

PN is also expected to enhance collagen formation and alleviate inflammation as part of the treatment for enlarged facial pores, and has been widely used for treatment of facial pores in South Korea since 2015.^14^ However, the details regarding the preparation, mode, and frequency of application of PN are unclear. It is essential to understand how cosmetic physicians use PN in clinical practice, including its application frequency and layering techniques, to optimize its efficacy. Given the lack of good direct preclinical and clinical evidence of the effectiveness of PN on enlarged facial pores, it would be helpful to know how cosmetic physicians uses PN and how they perceive its effectiveness. Therefore, the aim of this study was to assess cosmetic physicians’ current practices and their perceptions regarding the effectiveness of PN in treating enlarged facial pores.

## 2 MATERIALS AND METHODS

### 2.1 Survey development process

To gain insight into current practices and perceived effectiveness of PN, we reviewed previous studies.^8^, ^10^, ^11^, ^12^, ^13^, ^15^, ^16^, ^17^ The survey instrument was developed through face‐to‐face consultation interviews with expert cosmetic clinicians. Survey items were refined through direct discussions with other clinicians to compose the draft survey. A pilot study was conducted with a sample of seven cosmetic experts to test the draft survey and ensure its ease of use and external validity. Minor changes were made to the wording of survey questions to increase clarity based on the feedback received from the pilot study. The pilot sample consisted of cosmetic clinicians (*N* = 6) who were not included in the main study.

### 2.2 Survey content

These questions were designed to collect information on current practices and perceived effectiveness of PN for the treatment of enlarged facial pores. The survey was developed to distinguish three major causes of enlarged facial pores: (1) excessive sebum production, (2) reduced skin elasticity, and (3) acne.^2^

#### 2.2.1 Perceived effectiveness

The initial question sought information on clinician experience with PN usage, presented in a multiple‐choice format. Respondents selected from four options: “less than 10 cases,” “between 10 and 50 cases,” “between 50 and 100 cases,” and “more than 100 cases.” Respondents who chose “less than 10 cases” were excluded, as this selection was considered a surrogate measure for the inclusion criterion specifying relevant experience with PN.

If they had experienced more than 10 cases, clinicians were asked whether they use PN to treat enlarged facial pores for each of the three listed indications (excessive sebum production, reduced elasticity, acne). If they answered “yes” to each indication, they were prompted to answer a second question regarding the number of cases in which they have used PN for that indication. If they answered “no” to a specific indication, subsequent related questions were skipped.

For each indication, they were asked to rate the effectiveness of PN on a 4‐point scale ranging from “very ineffective” to “very effective.” They were also asked to provide their opinion on different proposed mechanisms of action of PN for the treatment of facial pores: (1) wound healing/regeneration, (2) alleviation of side effects after aesthetic procedures, (3) anti‐inflammation, (4) protection of the skin barrier, (5) hydration, (6) stabilization of sebum production, and (7) remodeling of the dermal matrix. For each of these mechanisms, respondents chose one of four options: (1) strongly agree, (2) agree, (3) disagree, and (4) strongly disagree.

To investigate how the clinicians apply PN for different indications, we asked the clinicians to indicate whether they would apply PN in the following situations: (1) patients with skin disease; (2) patients with sensitized skin due to aesthetic procedures; (3) patients with scar‐related acne; (4) patients with excessive sebum production; (5) patients with enlarged pores due to aging.

#### 2.2.2 Practice patterns

After that, respondents were asked about their current practice patterns of PN for treating enlarged facial pores, specifically regarding their use in combination with other devices or other injection therapies. They were provided with a list of devices, such as radiofrequency (RF), high‐intensity focused ultrasound, and laser, as well as a list of injectable treatments, including botulinum toxin (BoNT), hyaluronic acid, and poly‐lactic acid.

Finally, clinicians were asked about injection depth and frequency for the treatment of enlarged facial pores. They were also asked to report the proportion of cases of adverse events they observed, and were allowed to describe these adverse events in more detail if necessary.

### 2.3 Data collection

An online questionnaire was developed in an iterative process through several stages using SurveyMonkey (San Mateo, CA). The survey was distributed to the participants at the Korean Aesthetic Surgery & Laser Society Autumn Symposium 2023, held in Seoul, Republic of Korea, on September 10, 2023. Clinicians were allowed to complete the survey on their mobile devices. Each individual received a unique encrypted URL, ensuring that survey participants could only respond once. All data were encrypted, and all personally identifying information was removed.

All participants were provided with a consent form regarding the use of personal information, an agreement for its use, and consent to participate in the survey. The Institutional Review Board of Samsung Medical Center approved the protocol, study, and informed consent forms before enrollment (SMC‐2023‐08‐028‐002).

### 2.4 Statistical analysis

Categorical data are presented as proportions. Firstly, we conducted frequency analysis to understand the general characteristics of the study participants. Secondly, we used descriptive statistics and graphical representations to summarize the data. All statistical analyses were performed using R ver. 4.3.1 software (R Foundation for Statistical Computing, Vienna, Austria).

## 3 RESULTS

### 3.1 Baseline characteristics

Four hundred ninety‐seven clinicians participated in the study. Sixty‐one participants who had experienced fewer than 10 PN cases were excluded. An additional 29 participants were excluded due to incomplete data, ultimately resulting in 407 clinicians being included in final analysis. The participants in this study were predominantly aesthetic physicians and male, with 1–5 years of cosmetic procedure experience (Figure 1).

**FIGURE 1:** Characteristics of the 407 clinicians enrolled in the study.

### 3.2 Evaluating use and perceived effectiveness of PN for treating enlarged facial pores due to excessive sebum production

Among 407 respondents, 75.7% (308) answered they use PN to treat enlarged facial pores caused by excessive sebum production (Figure 2). Among them (*N* = 308), the majority of respondents (88.3%) used PN in combination with energy‐based devices, such as microneedle RF or non‐invasive RF. Additionally, over 70% of respondents used PN in combination with another injection therapy, mainly with BoNT (58.8%) (Figure 3A–C).

**FIGURE 2:** Clinician responses on the use of PN for facial pore enlargement caused by excessive sebum production, reduced elasticity, and acne.

**FIGURE 3:** PN procedure modalities for facial pore enlargement caused by excessive sebum excretion, reduced elasticity, and acne. (A) Combination of PN with other therapies. (B) Energy‐based devices. (C) Injection therapy.

The majority of respondents who used PN for facial pores enlarged by excessive sebum production agreed (78.2%) or strongly agreed (3.2%) with the efficacy of PN for this indication. Wound healing/promoting regeneration (81.2%) were most common mechanism selected for this indication, followed by alleviation of side effects after combined treatment (45.8%), hydration (41.2%), and protection of the skin barrier (38.3%) (Figure 4A,B).

**FIGURE 4:** Clinician's opinion of PN effectiveness for enlarged facial pores. (A) Level of effectiveness. (B) Perceived mechanism of action.

### 3.3 Evaluating clinicians’ use and perceived effectiveness of PN for treating enlarged facial pores due to reduced elasticity

In total, 87.7% (357 of 407 respondents) used PN to treat enlarged facial pores caused by reduced elasticity (Figure 2). Within this group (*N* = 357), the majority (88.5%) combined PN with energy‐based devices like microneedle RF or non‐invasive RF. About 80% of respondents used PN in combination with injection therapy, predominantly with BoNT (Figure 3A–C).

Among clinicians using PN for facial pores enlarged by reduced elasticity, the majority agreed (80.4%) or strongly agreed (3.4%) with the efficacy of PN for this indication. The primary mechanisms for PN in this indication were perceived to be wound healing/promoting regeneration (83.8%), followed by protection of the skin barrier (44.8%), alleviation of side effects after combined treatment (44.0%), and hydration (41.2%) (Figure 4A,B).

### 3.4 Evaluating clinicians’ use and perceived effectiveness of PN for treating enlarged facial pores due to acne

Among the 407 respondents, 72.2% (294) reported using PN to treat enlarged facial pores caused by acne (Figure 2). Within this group (*N* = 294), the majority of respondents (88.8%) combined PN with energy‐based devices, such as microneedle RF or non‐invasive RF. Additionally, 75.5% of respondents used PN in combination with injection therapy, primarily with BoNT (58.5%) (Figure 3A–C).

For clinicians using PN to treat enlarged facial pores related to acne, the majority (71.4%) agreed or strongly agreed (3.2%) with the efficacy of PN for this indication. The primary mechanisms for PN in this indication were perceived to be wound healing/promoting regeneration (82.3%), followed by alleviation of side effects after combined treatment (47.6%), protection of the skin barrier (41.5%), and anti‐inflammation (40.5%) (Figure 4A,B).

### 3.5 Clinicians’ agreement with suggested indications

87% of respondents reported using PN to treat enlarged pores due to aging. Also, 80.3% of respondents recommended PN for patients with skin sensitized by aesthetic procedures. Moreover, 77.9% of respondents reported utilizing PN for patients with scar‐related acne. PN was also applied in the treatment of patients with excessive sebum production (75.2%) and those with various skin diseases (68.3%) (Figure 5).

**FIGURE 5:** Clinicians’ agreement with suggested indications.

### 3.6 Current practice patterns

More than half of respondents typically used PN injections in the intradermal skin layer to treat enlarged facial pores. It was common clinical practice to inject PN in three to four sessions to treat enlarged facial pores. Furthermore, the distribution of patients across various age groups revealed diversity in the treatment of enlarged facial pores. The majority of patients were in their 30s and 40s (31.2% and 27.3%, respectively). Additionally, 24.2% of the patients were male (Figure 6). In this study, 95.0% of respondents reported rare adverse reactions, with the majority being mild and already documented in the package insert. The most prevalent adverse events were local injection reactions.

**FIGURE 6:** Current practice patterns.

## 4 DISCUSSION

To the best of our knowledge, this study is the first to investigate the current use patterns and perceived effectiveness of PN for enlarged facial pores among clinicians. As there is limited preclinical and clinical evidence on this topic, we conducted a survey of clinicians who have used PN in real‐world situations. This study provides practical information to guide the use of PN and inform further research.

We observed that a high proportion of cosmetic physicians used PN to treat enlarged facial pores caused by excessive sebum production, reduced elasticity, and/or acne. Approximately 80% of respondents reported that PN was “very effective” or “effective” in treating these indications. The majority of physicians utilized PN in combination with microneedle RF or BoNT to treat enlarged facial pores in this study.

In the survey, a considerable number of clinicians reported using PN as a treatment for facial pore enlargement attributed to excessive sebum production. The skin's ability to balance sebum is primarily associated with the stratum corneum, which consists of corneocytes and an intercellular lipid bilayer matrix.^18^ A reduction in the efficiency of the skin barrier results in changes to the sebum excretion rate. This rate reflects the amount of the sebum production and is closely related to the physiological activity of the sebaceous glands.^19^ PN supports both barrier organelles and structural scaffolds that aid in the proper accumulation of extracellular matrix.^12^ Therefore, the enhancement of the skin barrier through PN treatment could result from improvement of facial pores enlarged by excessive sebum production. Recently, there has been some discussion about methods for quantifying sebum levels.^20^ Further studies evaluating sebum excretion after PN injection are warranted.

The study found that a considerable number of clinicians used PN and agreed with its effectiveness for treating enlarged facial pores caused by reduced elasticity. Earlier studies confirmed that PN plays a role in collagen synthesis, reporting an increase in collagen I synthesis in vitro via human fibroblasts in primary cultures.^21^ Recently, several clinical studies have investigated the efficacy of PN, with most showing promising results regarding collagen synthesis, a key factor in improving skin elasticity.^15^, ^22^ This was evidenced by collagen composition assessments using ultrasound and a three‐dimensional camera in patients treated with PN.^22^ In addition, a case report demonstrated significant improvements in facial pore size and skin thickness.^14^ These findings help to explain the mechanism behind PN's usefulness in treating facial pore enlargement associated with reduced elasticity, as described in our analysis.

We observed that 72.2% of clinicians used PN to treat acne‐induced facial pore enlargement, with 76.8% of these clinicians reporting its effectiveness. Although the presence of acne is associated with enlarged facial pores, acne severity does not correlate with increased pore size.^23^ However, acne and facial pores are linked as open comedones tend to reside in the pores.^23^ Previous studies have identified the activation of proinflammatory cytokines in the skin of patients with acne.^24^ A previous in vitro study demonstrated that PN inhibits the inflammatory response of interleukin‐1β by decreasing the expression of pro‐inflammatory cytokines, such as matrix metalloproteinases, iNOS, cyclooxygenase‐2, and nitric oxide production.^25^ This sheds light on the potential of PN as an anti‐inflammatory treatment for acne‐induced facial pore enlargement.

The survey results showed that clinicians widely agree on the effectiveness of PN for various other indications. These indications were prioritized as follows: patients with aging‐related facial pore enlargement, patients with sensitized skin resulting from aesthetic procedures, patients with scar‐related acne, patients experiencing excessive sebum production, and patients with other skin diseases.

The diverse indications for PN align with its underlying mechanisms. PN not only fills the contracted or depressed space but also enhances tissue regeneration, effectively reducing wrinkles and rejuvenating the aging face.^14^ PN is beneficial for patients with skin irritation and dryness due to its hydrating properties, particularly when the skin's scaffolding is weakened.^26^ It also exhibits anti‐inflammatory effects, reducing proinflammatory cytokines involved in the pathogenesis of acne and skin diseases.^25^ Moreover, PN contributes to skin barrier protection through collagen synthesis,^15^ promoting balanced sebum production. This approach highlights the versatility of PN in addressing various skincare needs.

Our analysis revealed that the most frequent energy‐based device treatment used in combination with PN was microneedle RF. Recently, microneedle RF has emerged as an effective treatment for significantly reducing pore size while avoiding the side effects of laser therapy, such as indirect damage to the epidermis (e.g., burns).^27^ This is achieved by microneedle RF through the creation of coagulation canals within the dermis via needle tunneling,^28^ stimulating the formation of new collagen and resulting in tightened and rejuvenated skin.^29^ Therefore, RF is responsible for stimulating collagen fibers when combined with PN. Additionally, microneedle RF creates an oscillating electrical current, which induces vibration and collisions of charged molecules, leading to heat production.^30^ It is expected that simultaneous thermal stimulation increases the collagen synthesis associated with PN.^31^ PN can also relieve skin dryness,^11^ which is a common side effect of RF treatment. The combined use of RF with PN is thus thought to produce synergistic effects.

Around 50% of surveyed clinicians used PN in combination with BoNT as an injection therapy to treat enlarged facial pores. BoNT is well known for significantly reducing pore size.^32^ Although the mechanism through which BoNT reduces sebum production is not entirely clear, studies have revealed that sebaceous glands express nicotinic acetylcholine receptor α7 and release acetylcholine locally, potentially influencing sebum production. Through this pathway, BoNT is believed to decrease sebum production by inhibiting cholinergic signaling.^33^ Furthermore, the neuromodulatory effects of BoNT on arrector pili muscles may also contribute to decreased sebum excretion.^34^

Therefore, BoNT is expected to induce a pore‐contracting effect through its inherent sebum‐regulating function and increased skin tension caused by mechanical damage from intradermal injections.^32^, ^33^, ^34^ The mechanisms of BoNT and PN do not overlap, so the combination of BoNT with PN for enlarged pore treatment seems like the optimal combination.

In this study, we conducted a survey to investigate clinicians’ current practices and perceived effectiveness when using PN to treat enlarged facial pores. While this survey offered efficient data collection and broad coverage, several limitations must be acknowledged. These include that the participants were exclusively from the Republic of Korea, which may limit the generalizability of the findings. There is also the possibility of misunderstanding or biased responses due to the wording of the questions. Despite these limitations, this study provides a comprehensive overview of PN use in treating enlarged facial pores. The aim was to enhance the understanding and effective utilization of injectable PN among cosmetic physicians.

## 5 CONCLUSIONS

In summary, cosmetic physicians in the Republic of Korea have used PN in the treatment of enlarged facial pores caused by excessive sebum production, reduced elasticity, and acne. Most of these clinicians agreed that PN had an effect on enlarged facial pores. These findings support the idea that using PN for enlarged facial pores treatment can be beneficial.

## CONFLICT OF INTEREST STATEMENT

H.C., K.Y., Y.J.P., H.J.P., S.M.O., G.H.J., and G.C.R. are on the advisory board of PharmaResearch Co. Ltd. (Republic of Korea).

## Data Availability

The data that support the findings of this study are available on request from the corresponding author. The data are not publicly available due to privacy or ethical restrictions.
